# A Benign and Malignant Breast Tumor Classification Method via Efficiently Combining Texture and Morphological Features on Ultrasound Images

**DOI:** 10.1155/2020/5894010

**Published:** 2020-10-01

**Authors:** Mengwan Wei, Yongzhao Du, Xiuming Wu, Qichen Su, Jianqing Zhu, Lixin Zheng, Guorong Lv, Jiafu Zhuang

**Affiliations:** ^1^College of Engineering, Huaqiao University, Quanzhou 362021, China; ^2^School of Medicine, Huaqiao University, Quanzhou 362021, China; ^3^Collaborative Innovation Center for Maternal and Infant Health Service Application Technology, Quanzhou Medical College, Quanzhou, China; ^4^The First Hospital of Quanzhou, Fujian Medical University, Quanzhou 350005, China; ^5^Department of Medical Ultrasonics, The Second Affiliated Hospital of Fujian Medical University, Quanzhou 362000, China; ^6^Quanzhou Institute of Equipment Manufacturing, Haixi Institutes, Chinese Academy of Sciences, 362216 Quanzhou, China

## Abstract

The classification of benign and malignant based on ultrasound images is of great value because breast cancer is an enormous threat to women's health worldwide. Although both texture and morphological features are crucial representations of ultrasound breast tumor images, their straightforward combination brings little effect for improving the classification of benign and malignant since high-dimensional texture features are too aggressive so that drown out the effect of low-dimensional morphological features. For that, an efficient texture and morphological feature combing method is proposed to improve the classification of benign and malignant. Firstly, both texture (i.e., *local binary patterns* (LBP), *histogram of oriented gradients* (HOG), and *gray-level co-occurrence matrixes* (GLCM)) and morphological (i.e., shape complexities) features of breast ultrasound images are extracted. Secondly, a *support vector machine* (SVM) classifier working on texture features is trained, and a *naive Bayes* (NB) classifier acting on morphological features is designed, in order to exert the discriminative power of texture features and morphological features, respectively. Thirdly, the classification scores of the two classifiers (i.e., SVM and NB) are weighted fused to obtain the final classification result. The low-dimensional nonparameterized NB classifier is effectively control the parameter complexity of the entire classification system combine with the high-dimensional parametric SVM classifier. Consequently, texture and morphological features are efficiently combined. Comprehensive experimental analyses are presented, and the proposed method obtains a 91.11% accuracy, a 94.34% sensitivity, and an 86.49% specificity, which outperforms many related benign and malignant breast tumor classification methods.

## 1. Introduction

Breast cancer is a common cause of death for women worldwide. According to the global cancer statistics 2018 [1], the incidence and mortality of cancer in China rank the first in the world, among which the incidence of breast cancer is the highest among women and the mortality rate ranks the fifth. Early detection, early diagnosis, and early treatment are the key to improve the recovery rate of breast cancer and reduce the mortality rate [2]. Therefore, it is desired to develop an effective benign and malignant breast tumor classification method.

Commonly, texture and morphological features of breast ultrasound images are used to analyze the benign and malignant of tumors. The straightforward approach is to rely on high-level and experienced radiologists to judge the benign and malignant of tumors by manually analyzing the texture and morphological features in images [3]. However, the proportion of each feature in the diagnosis in the comprehensive judgment is likely to lead to poor objectivity and repeatability of the diagnosis results due to different doctors' technology and experience. Moreover, ultrasound images themselves also have the disadvantages of high noise and low resolution, which greatly limit the accuracy of artificial ultrasonic detection.

Another straightforward approach is to train classifiers based on texture and morphological features by a computer for classifying benign and malignant tumors automatically to overcome the subjectivity of manually ultrasound image analysis [4]. There are two primary methods of computer automatic analysis. One method is to utilize single features (one of texture features and morphological features [5–8]) with single classifier for computer modeling of breast images. However, this method [5–8] does not fully consider the complementarity of features, and the accuracy of classification is restricted. Another method utilizes multiple features (texture and morphological features) with single classifier [9–12] to take advantage of the complementarity between texture and morphological features. Nevertheless, the direct combination of multiple features will affect the performance of classification such as high-dimensional texture features are too aggressive so that drown out the effect of low-dimensional morphological features [13]. Single classifier cannot solve this problem. Therefore, the main purpose of this article is to effectively combine texture and morphological features to improve the classification performance.

For that, a benign and malignant breast tumor classification method via efficiently combing texture and morphological features is proposed.  Figure 1 shows an overview of the proposed method. One can see that two different classifiers are used to train texture and morphological features, respectively, in the proposed method. Firstly, three texture features (*local binary patterns* (LBP) [14], *histogram of gradients* (HOG) [15], *gray-level co-occurrence matrixes* (GLCM) [16]) and three morphological features (compactness, elliptical compactness, and radial distance spectrum) are extracted from 448 collected breast ultrasound images which have been denoised and equalized. Then, the dimensions of texture features are reduced by PAC. Secondly, using *support vector machine* (SVM) [17] classifier and *naive Bayes* (NB) [18] classifier to, respectively, learn texture features and morphological features. SVM is already a high-dimensional parametric classifier. If one wants to combine multiple classifiers, according to Occam's razor [19], it is reasonable to select a low-dimensional nonparametric classifier to control the parameter complexity of the entire classification system. Thirdly, the outputs of the two classifiers are weighted fused to obtain the final classification result.

This paper is an extension of our preliminary works [20, 21], which improves both methodology and experimental analysis. The contributions of this paper can be summarized as follows. (1) A novel method is proposed to effectively combine multiple features and multiple classifiers to improve the benign and malignant breast tumor classification performance. Specifically, in order to avoid the sharp increase in parameter complexity caused by using multiple classifiers, a nonparameterized NB classifier trained on low-dimensional morphological features is designed to cooperate with a parameterized SVM classifier trained on high-dimensional texture features. (2) Comprehensive experimental analyses are presented to verify the advantage of the proposed method, including data preprocessing, dimension reduction, single feature with single classifier, multiple features with single classifier, and effectively combining multiple features and multiple classifiers.

The rest of this paper is structured as follows.  Section 2 introduces the related work.  Section 3 describes the feature extraction, the experimental details, and the collected breast ultrasound image dataset.  Section 4 presents the experimental results to analyze the effectiveness of the proposed method.  Section 5 concludes this paper.

## 2. Related Work

With the progress of computer technology, medical imaging technology has been greatly developed. It has become a trend to use the computer to classify breast ultrasound images automatically. In this section, an overview of based on hand-crafted features and deep-learned feature methods for breast tumor classification is presented.

### 2.1. Hand-Crafted Features for Breast Tumor Classification

In breast ultrasound images, the traditional breast tumor classification technology mainly includes the following four steps [22, 23]: image preprocessing, image segmentation, feature extraction, and tumor classification. Among them, feature extraction is the main task of breast tumor classification, which has a great impact on the classification results [24]. Texture (i.e., LPB [14], HOG [15], and GLCM [16]) and morphological (i.e., shape complexities) which called hand-crafted features are the key to analyze breast ultrasound images. The hand-crafted feature-based breast tumor classification methods can be roughly divided into two categories.

Firstly, the most common method is to model the breast ultrasound images using single features (one of texture features and morphological features) with single classifier [5–8]. For example, Pomponiu et al. [5] filtered tumors and normal areas based on the histogram of oriented gradients (HOG) descriptor and used SVM to classify the recognized tumors. Mohamed et al. [8] used a superresolution method to preprocess ultrasound images and evaluated the performance of five texture features.

Secondly, many methods are to model the breast ultrasound images using multiple features (texture features and morphological features) with single classifier [9–12]. For example, Menon et al. [10] extracted the textural, morphological, and histogram features of tumor ultrasound images and used SVM to classify tumors. Gonzelezluna et al. [12] extracted 41 morphological features and 96 texture features to analyze the classification effects of 7 classifiers.

In addition, SVM [17], NB [18], *k-nearest neighbor* (KNN) [25], *decision tree* (DT) [26], *linear discriminant analysis* (LDA) [27], and other classifiers are commonly used in hand-crafted feature methods. These classifiers can be divided into two categories: parameterized classifiers and nonparameterized classifiers. Generally, in the process of classification, the calculation of parameterized classifier is complicated which needs to train repeatedly to obtain the best parameters, but this kind of classifier has strong generalization ability on small data sets, such as SVM [17] and KNN [25]. The nonparameterized classifier does not introduce additional parameter complexities although it has poor generalization ability on small data sets, such as NB [18]. When combining multiple features with different classifiers, using two parameterized classifiers will make the training model too complicated, while two nonparameterized classifiers lack strong discrimination learning ability [19]. Therefore, a parameterized classifier with a nonparameterized classifier is proposed to combine multiple features.

### 2.2. Deep-Learned Features for Breast Tumor Classification

Deep neural networks, powered by advances in computing capability and very large annotated datasets, have achieved revolutionary breakthroughs in computer vision [28]. CNN [29] is the most basic method for classification of breast tumors by deep-learned features. For example, both Zhou et al. [29] and Qi et al. [30] used CNN to extract image features and classify benign and malignant tumors automatically. Other deep-learned features are also applied to the classification of breast tumors. Choi et al. [31] evaluated a computer-aided diagnostic system that combines three deep learning models (Fully Convolutional Network (FCN) [32], AlexNet [33], and GoogLeNet [34]) by comparing the diagnostic results of the doctors and computer.

## 3. Materials and Methods

### 3.1. Data Acquisition and Preprocessing

Although there are indeed some breast ultrasound databases, they are not easy to obtain for protecting the privacy of patients. Therefore, a new dataset of breast ultrasound images is collected in Quanzhou First Hospital in Fujian, China, since the public ultrasound images are not easy to obtain and may infringe the patient's privacy. All the images were collected by PHILIPS iu22, PHILIPS iu Elite, and other color ultrasound diagnostic devices with the probe frequency of 12 MHz from 2018 to 2019. The imaging parameters of the ultrasound device were adjusted by radiologists. The images are used with the consent of the relevant patients.  Figure 2 shows same examples of the collected ultrasound images.

Cases with previous breast surgery history, poor image quality, and incomplete clinical data were removed, and 448 breast ultrasound images were finally obtained. Among them, 184 are benign tumors, and 264 are malignant tumors. All cases underwent biopsy. According to the definitions of assessment categories in breast imaging reporting and data system (BI-RADS) [3, 35], the final assessment of 448 solid breast tumors on the basis of ultrasound findings is category 2, consider benign changes, for 43 tumors (9.6%); category 3, probably benign tumors, for 50 tumors (11.2%); category 4a, low probability of malignancy, for 91 tumors (20.3%); category 4b, median probability of malignancy, for 77 tumors (17.2%); category 4c, high probability of malignancy, for 66 tumors (14.7%); category 5, highly suspicious of malignancy, for 106 tumors (23.7%); and category 6, malignant tumors, for 15 tumors (3.3%). The collected data covers all tumor categories.  Figure 3 shows the distribution of the collected images. For each breast ultrasound image, the *region of interest* (ROI) and outline of tumors are manually annotated by a high-level professional radiologist with more than 10 years of experience. And the annotated results are verified by another experienced radiologist.

The edges of all the images are removed at first. At the same time, due to the presence of speckle noise and low contrast in ultrasound imaging, the ability of the computer to fully extract texture and morphological features will be limited. For this, all the images are denoised by *speckle reducing anisotropic diffusion* (SRAD) filter [10]. Then, the denoised images are equalized using histogram. The result after using SRAD filter and histogram to denoise and equalize the breast ultrasound images is shown in Figure 4. Compared with the original images, the denoised and equalized images show better resolution and contrast.

### 3.2. Feature Extraction and Selection

#### 3.2.1. Feature Extraction

The feature extraction of breast ultrasound image is a key step in the classification of benign and malignant breast tumors. By extracting a large number of features from ultrasound images and quantifying major diseases such as tumors, the problem of quantitative evaluation of tumor heterogeneity can be effectively solved. It is of certain significance to introduce texture features for tumor analysis since there are significant differences in internal echoes and boundary echoes of typical benign and malignant tumors in ultrasound imaging. Therefore, the local binary patterns (LBP) [14], histogram of oriented gradients (HOG) [15], and gray-level co-occurrence matrixes (GLCM) [16] features are extracted for classifying. At the same time, benign and malignant tumors often show differences in morphology. It is generally believed that benign tumors are of regular shape, mostly round or oval shape, and the tumor contour itself is relatively smooth. But malignant tumor is on the contrary. Therefore, compactness, elliptical compactness, and radial distance spectrum are extracted to reflect the complexity of tumor contour.

*(1) Texture Features*. The LBP [14] is an operator used to describe local texture features of the image, which has obvious advantages such as rotation invariance and gray invariance. The LBP [14] operator is defined as a 3 × 3 window. An ordered 8-bit binary number is generated by comparing the size of the central pixel value with the surrounding pixel value (usually converted to LBP [14] code, which is 256 decimal), expressed as follows:

(1) $$\begin{array}{c} \text{LBP}\left(x,y\right)=\overset{8}{\underset{p=1}{\sum }}2^{p‐1}s\left(i_{p}-i_{c}\right),\\ s\left(x\right)=\left\{\begin{array}{c} 1\text{ if }x\geq 0\\ 0\text{ else} \end{array}\right., \end{array}$$

where *i* is the gray value of the center pixel (*x*, *y*), *p* is the number of the adjacent pixel, *i*_*p*_ is the gray value of the adjacent pixel, and s(*x*) is the symbolic function.

The HOG [15] forms the feature by calculating and statistics the histogram of gradient direction in the local area of the image. Firstly, the image is Gamma corrected, and the gradient of each pixel is calculated. Secondly, the image is divided into 32 × 32 pixel cells in this paper, and the histogram of gradient of each cell is counted to form a descriptor. Finally, every 2 × 2 cell is concatenated to form a block, and then, all blocks are concatenated to get the HOG [15] feature descriptor.

The GLCM [16] extracts the relationship between the pixel pairs. In this paper, the grayscale level is set to 64. The distance between pixels is adjusted within the range of [1, 10], and the relationship between pixels with a certain distance is calculated from four directions (0, 45, 90, 135). Finally, 40 different matrices are obtained from each image. The energy, contrast, correlation, and homogeneity are extracted from matrices to reflect the roughness of the texture, the local variation, and the uniformity of the gray distribution of the image.

*(2) Morphological Features*. Morphological features are obtained by calculating the compactness (equation (2)), the elliptic compactness (equation (3)), and the mean and variance of the radial distance spectrum (equation (4)) of the tumor. The tumor has the potential to be malignant if the shape of the tumor looks like irregular lobules, rather than just round or oval [8].

Compactness measures the similarity between the shape of a breast tumor and its fitting circle. The closer the compactness value is to 1, the less likely the tumor is to be malignant, expressed as follows:

(2) $$\begin{array}{c} C=\frac{A}{4\pi L^{2}}, \end{array}$$

where *A* represents the area of the tumor and *L* is the perimeter of the breast tumor contour.

The elliptic compactness is the ratio of the circumference of the fitting ellipse to the circumference of the original tumor contour. It is negatively correlated with the degree of malignancy of the tumor. The elliptic fitting method is to find an ellipse for a given set of tumor contour points and make it as close as possible to these contour points. More generally, the contour points of the tumor are fitted with the elliptic equation as the model so that a certain elliptic equation can satisfy these points as far as possible, and each parameter of the elliptic equation is obtained. Here, used the least square method proposed by Fitzgibbon et al. [36] for ellipse fitting. The effect of ellipse fitting is shown in Figure 5. The blue line is the contour of the tumor, and the red line is the fitting ellipse. According to the fitting ellipse obtained, the features are calculated as follows:

(3) $$\begin{array}{c} EC=\frac{\pi \left(a+b\right)}{D}, \end{array}$$

where *a* represents the semimajor axis of the fitting ellipse, *b* is the semiminor axis of the fitting ellipse, and *D* is the perimeter of the breast tumor contour.

Radial distance spectrum method quantified the degree of tumor margin roughness by statistical and analyzing the radial distance from each point on the tumor margin to the tumor center. In this paper, Fourier transform is applied to the obtained radial distance spectrum, and its logarithm is taken to obtain the logarithmic amplitude spectrum of radial distance. Finally, the mean and variance of harmonic components in the logarithmic amplitude spectrum are taken as characteristic parameters. Radial distance can be calculated as follows:

(4) $$\begin{array}{c} D\left(t\right)=\sqrt{{\left(p_{t}-x_{0}\right)}^{2}+{\left(q_{t}-y_{0}\right)}^{2}}, \end{array}$$

where the tumor edge points are denoted as *P*_*t*_(*p*_*t*_, *q*_*t*_) and the center point is denoted as (*x*_0_, *y*_0_).

#### 3.2.2. Feature Selection

In this paper, the *principal component analysis* (PCA) [37] is used to reduce the dimension of extracted texture features in order to speed up the training and testing time and improve the efficiency of the proposed method.

### 3.3. Experiments

#### 3.3.1. Experimental Setup

It is well-known that texture and morphological features are complementary in the ultrasound image. However, the classification ability via combining texture and morphological features directly will be limited because of the aggressiveness of high-dimensional texture features. For that, a classification method for benign and malignant breast tumor via efficiently combining texture and morphological features is proposed in this paper. The specific process is shown in Figure 1. The collected breast ultrasound images are randomly divided into training set (80%) and test set (20%); then, all images are preprocessed. Three texture features (i.e., LBP [14], HOG [15], and GLCM [16]) and three morphological features (compactness, elliptical compactness, and radial distance spectrum) are extracted and normalized. The dimensions of the extracted texture features are reduced by PCA [37]. On the account of high-dimensional texture features can easily affect low-dimensional morphological features in the single classifier, support vector machine (SVM) [17] and naive Bayes (NB) [18] classifiers are used to learn texture features and morphological features, respectively, in this paper. SVM is already a high-dimensional parametric classifier. If one wants to combine multiple classifiers, according to Occam's razor [19], it is reasonable to select a low-dimensional nonparametric classifier to control the parameter complexity of the entire classification system. Finally, the classification scores of the two classifiers are weighted fused (equation (5)) to obtain the final classification result:

(5) $$\begin{array}{c} S_{c}\left(\lambda \right)=S_{\text{SVM}}\times \lambda +S_{\text{NB}}\times \left(1-\lambda \right), \end{array}$$

where *λ* represents the weight, ranging from 0 to 1; *S*_SVM_ is the score of malignant classification output by SVM classifier; *S*_NB_ is the score of malignant classification output by NB classifier; and *S*_*c*_(*λ*) represents the weighted fusion of the classification scores of two classifiers (SVM and NB) and its values between 0 and 1. When the value of *S*_*c*_(*λ*) is greater than or equal to 0.5, the tumor is considered malignant; when the value of *S*_*c*_(*λ*) is less than 0.5, the tumor is considered benign.

Comprehensive experimental analyses are presented, and the experiment is divided into three parts to compare and analyze the advantages of the proposed method. In the first part, the classification performance of using single features with single classifier is evaluated and compared. In the second part, the classification performance of using multiple features with single classifier is evaluated and compared. In the third part, the classification performance of using multiple features with multiple classifiers is evaluated and compared. Another three classifiers (k-nearest neighbor (KNN) [25], decision tree (DT) [26], and linear discriminant analysis (LDA) [27]) are used to analyze the three extracted texture features and three morphological features in order to verify the superiority of the proposed method. The methods of analyzing features include single features and combined multiple features.

In this work, the parameters of each classifier are optimized to improve the classification performance. In SVM [17], the radial basis function is used as the kernel function, and the mesh search method is used to perform the 5-fold cross-validation to automatically find the optimal penalty factor *c* and the kernel parameter *g*. The number of neighbors in KNN [25] is set to 5.

#### 3.3.2. Evaluation Criterion

The classification performance is quantitatively measured by accuracy, sensitivity, and specificity [38]. In addition, the receiver operating characteristic (ROC) curve analysis is used to evaluate the performance of classifiers. The area under the curve (AUC) is calculated based on the ROC to measure the ability of features to distinguish benign and malignant tumors.

## 4. Results and Discussion

### 4.1. Experimental Results

The result of the proposed method is verified through a comparison in the following. Support vector machine (SVM) [17] and naive Bayes (NB) [18] classifiers are used to effectively learn texture features (local binary patterns (LBP) [14], histogram of gradients (HOG) [15], gray-level co-occurrence matrixes (GLCM) [16]) and morphological features (compactness, elliptical compactness, and radial distance spectrum), respectively, in this paper. In order to show the superiority of the proposed method, this paper compares it with the related methods [5, 7, 8, 10, 12]. The experiments are mainly completed on Matlab 2017b.

It can be seen from Table 1 that the hand-crafted feature method can learn a small sample well to get a better classification effect. In addition, the experimental results show that the classification performance of multiple features is often better than single feature, and our method takes full advantage of the complementarity of texture and morphological features to get the better performance than single classifier. The performance of our method is superior to other related methods, with the accuracy of 91.11%, the sensitivity of 94.34%, and the specificity of 86.49%. The effective combination of multiple features and multiple classifiers can effectively improve the classification of benign and malignant breast tumors.

### 4.2. Discussion

In order to prove the effectiveness of the proposed method, the following analysis and discussion are carried out. Another three classifiers (k-nearest neighbor (KNN) [25], decision tree (DT) [26], and linear discriminant analysis (LDA) [27]) with SVM [17] and NB [18] are used to analyze the three extracted texture features (LBP [14], HOG [15], GLCM [16]) and three morphological features (compactness, elliptical compactness, and radial distance spectrum). The experimental analysis will be carried out from three subsections as follows.

#### 4.2.1. Experiments Based on Classification Methods Using Single Features with Single Classifier

Based on LBP [14], HOG [15], GLCM [16] texture features, fused texture features, and morphological features, the detailed data of sensitivity, specificity, and accuracy of model prediction are shown in Table 2.

Compared with the classification results of different texture features in Table 2, the classification results based on the fused texture features are the best, with the accuracy reaching 86.67%, the sensitivity reaching 92.45%, and the specificity reaching 78.38%. The second best feature is LBP [14], which achieves 85.56% in accuracy, 86.79% in sensitivity, and 83.78% in specificity. The accuracy of HOG [15] feature is 81.11%, the sensitivity is 84.91%, and the specificity is 75.68%. The accuracy of GLCM [16] is 78.89%, the sensitivity is 92.45%, and the specificity is 59.46%. For morphological features, the accuracy is 81.11%, the sensitivity is 69.81%, and the specificity is 97.30%.

By comparing the classification results of different classifiers in Table 2, the classification results of SVM [17] classifier are generally higher than those of other classifiers, with the accuracy reaching 86.67%, the sensitivity reaching 92.45%, and the specificity reaching 78.38%. The second is KNN [25] classifier, with accuracy of 84.44%, sensitivity of 84.91%, and specificity of 83.08%. The NB [18] classifier achieves 81.11% in accuracy, 69.81% in sensitivity, and 97.30% in specificity. The accuracy of LDA [27] classifier is 75.56%, the sensitivity is 60.38%, and the specificity is 97.30%. The accuracy of DT [26] classifier can reach 72.22%, the sensitivity is 73.58%, and the specificity is 60.27%.

By comparing the experimental results in Table 2, the best results of the single feature and single classifier classification methods are the fused texture features (LBP+HOG+GLCM) with SVM classifier. However, the complementarity of features is not fully considered to restrict the accuracy of classification in these methods of using single features with single classifier.

#### 4.2.2. Experiments Based on Classification Methods Using Multiple Features with Single Classifier

Multiple features provide a good way to identify benign and malignant tumors well [39] by considering the complementarity of texture and morphological features. Therefore, the classification method based on multiple features with single classifier is analyzed and discussed experimentally. The accuracy, sensitivity, and specificity are shown in Table 3.

Compared with the different combination of multiple features (texture features and morphological features) with single classifier (SVM and LDA), the classification result of the method using the fused texture features (LBP+HOG+GLCM) and morphological features with SVM classifier is the best. The accuracy, sensitivity, and specificity are 87.78%, 88.68%, and 86.49%, respectively. From the analysis of the experimental results in Tables 2 and 3, it can be concluded that the classification result is not ideal, although the method of multiple features with single classifier which straightforward combining texture features and morphological features have considered the complementarity of texture features and morphological features. This is because that the method of straightforward combining multiple features with single classifier has not consider the aggressiveness of high-dimensional texture features to low-dimensional morphological features.

#### 4.2.3. Experiments Based on Classification Methods Using Multiple Features with Multiple Classifiers

Based on the above analysis, the method of using SVM classifier and NB classifier working on texture and morphological features, respectively, is proposed in order to exert the discriminative power of texture features and morphological features. SVM is already a high-dimensional parametric classifier. If one wants to combine multiple classifiers, according to Occam's razor [19], it is reasonable to select a low-dimensional nonparametric classifier to control the parameter complexity of the entire classification system. The accuracy, sensitivity, and specificity are shown in Table 4.

From the analysis of the experimental results in Tables 3 and 4, it can be concluded that the proposed method of using SVM and NB classifier to effectively combine texture and morphological features has fully considered the complementarity of texture and morphological features and eliminates the aggressive of high-dimensional texture features to low-dimensional morphological features. The proposed methods are 3.33% and 5.66% higher than the method of using SVM [17] to directly combine texture and morphological features in the accuracy and sensitivity, respectively. At the same time, the accuracy of the proposed method is about 4.44% higher than the highest accuracy of single feature. The ROC curves of the three methods in Table 4 are shown in Figure 6. The AUC of the method based on texture feature and SVM [17] classifier reached 0.9118. The AUC based on morphological features and NB [18] classifier method reached 0.9174. The AUC of the proposed method is 0.9225. The final classification result of the proposed method is obtained from the weighted fused of the classification scores of SVM [17] and NB [18] classifiers as shown in equation (5).  Figure 7 shows the weight analysis of weighted fusion. When the weight is set from 0.6 to 0.9, the proposed method performs well. Among them, the accuracy is the highest when the weight is 0.8, and both sensitivity, specificity, and AUC are taken into account.

#### 4.2.4. Effect Analysis of Image Preprocessing and Feature Selection

To confirm that denoising and equalization have an auxiliary effect on classification of ultrasound image, the classification experiment is also performed using images without denoising and equalization, and the two results are compared. Due to the noise and contrast of the image that have little effect on the morphological features, this paper compares the experiments that only extract the texture features. The SVM classifier with the best classification performance is preprocessed to analyze the texture features. As shown in Table 5, preprocessing helps extract more useful texture features from images, efficiently improving accuracy.

The dimension of texture feature extracted for the first time is too large. The eigenvector matrix can be reduced by using PCA to retain the most effective features. As can be seen from Table 6, after dimension reduction of texture features, the time required for testing is greatly reduced, which improves efficiency of the whole classification method. Dimension reduction reduces the training time to 0.0135 s, 1/26 of the training time before dimension reduction.

## 5. Conclusion

In this paper, an efficient texture and morphological feature combining method is proposed to improve the classification performance of benign and malignant tumors in ultrasound imaging. Firstly, the texture features (i.e., local binary patterns (LBP), histogram of oriented gradients (HOG), and gray-level co-occurrence matrixes (GLCM)) and morphological features (i.e., compactness, elliptical compactness, and radial distance spectrum) are extracted from the collected 448 breast tumor ultrasound images after denoised and equalized. Secondly, support vector machine (SVM) and naive Bayes (NB) classifiers are used to learn texture features and morphological features, respectively, since high-dimensional texture features can easily affect low-dimensional morphological features in the single classifier. Finally, the classification scores of the two classifiers are weighted fused to obtain the final classification result. The low-dimensional nonparameterized NB classifier is effectively control the parameter complexity of the entire classification system combine with the high-dimensional parametric SVM classifier. Comprehensive experimental analyses are presented to verify the effectiveness of the proposed method that another three classifiers (i.e., k-nearest neighbor (KNN), decision tree (DT), and linear discriminant analysis (LDA)) are used to analyze the three extracted texture features and three morphological features in order to verify the superiority of the proposed method. The methods of analyzing features include single features and combined multiple features. Experimental results show that the proposed method has the best accuracy, sensitivity, and specificity. This provides a rapid, low-cost, and repeatable diagnostic method for the ultrasound examination of breast tumors and has certain feasibility and good robustness.

## Figures and Tables

**Figure 1:** A benign and malignant breast tumor classification method via efficiently combining textural and morphological features. ∑ represents the weighted fusion of the classification scores of the two classifiers (i.e., SVM and NB).

**Figure 2:** Samples of ultrasound images of breast tumors classified according to BI-RADs standard: (a, b) are benign tumors and (c, d) are malignant tumors. Benign tumors are usually well-defined and round or oval in shape. Malignant tumors are usually poorly defined and irregular with lobules.

**Figure 3:** Histogram distribution of 448 breast ultrasound images used for texture and morphological analysis.

**Figure 4:** The result after using SRAD filter and histogram to denoise and equalize the breast ultrasound images: (a) shows the original image, (b) shows the denoised image, and (c) shows the result after equalization.

**Figure 5:** The examples of the fitting ellipse that transformed from breast tumor contour: (a, b) malignant tumor and (c, d) benign tumor.

**Figure 6:** The ROC curve of different combinations of texture and morphological features with different classifiers.

**Figure 7:** The classifier weighted fusion analysis diagram.

**Table 1:** The performance comparison of our method and multiple related methods.

Method		Evaluation (%)		
		Accuracy	Sensitivity	Specificity
Single feature with single classifier (SFSC)	Pomponiu et al. [5]	81.11	84.91	75.68
	Biswas et al. [7]	75.56	67.92	86.49
	Mohamed et al. [8]	84.44	84.91	83.78

Multiple features with single classifier (MFSC)	Menon et al. [10]	87.78	88.68	86.49
	Gonzelezluna et al. [12]	86.67	88.68	83.78

Multiple features with multiple classifiers (MFMC)	Our method	91.11	94.34	86.49

**Table 2:** The classification results based on the methods of single features with single classifier.

Method		Evaluation (%)		
Feature	Classifier	Accuracy	Sensitivity	Specificity
LBP	SVM [17]	85.56	86.79	83.78
	KNN [25]	84.44	84.91	83.78
	DT [26]	66.33	58.49	81.08
	LDA [27]	74.44	77.36	70.27

HOG	SVM [17]	81.11	84.91	75.68
	KNN [25]	61.11	100.00	5.41
	DT [26]	67.78	67.92	67.57
	LDA [27]	70.00	75.47	62.16

GLCM	SVM [17]	78.89	92.45	59.46
	KNN [25]	65.56	75.47	51.35
	DT [26]	71.11	77.36	62.16
	LDA [27]	74.44	84.91	59.46

LBP+HOG+GLCM	SVM [17]	86.67	92.45	78.38
	KNN [25]	64.44	100.00	13.51
	DT [26]	72.22	73.58	70.27
	LDA [27]	75.56	84.91	62.16

Morphological	SVM [17]	75.56	67.92	86.49
	NB [18]	81.11	69.81	97.30
	LDA [26]	75.56	60.38	97.30

**Table 3:** The classification results based on the methods of multiple features with single classifier.

Features	Evaluation (%)	Classifier	
		SVM	LDA
LBP+ morphological	Accuracy	80.00	76.67
	Sensitivity	79.25	75.47
	Specificity	81.08	78.38

HOG+ morphological	Accuracy	83.33	72.22
	Sensitivity	81.13	71.70
	Specificity	86.48	72.97

GLCM+ morphological	Accuracy	80.00	80.00
	Sensitivity	69.81	81.13
	Specificity	94.59	78.38

LBP+HOG+GLCM+ morphological	Accuracy	87.78	76.67
	Sensitivity	88.68	75.47
	Specificity	86.49	78.38

**Table 4:** The classification results based on the method of multiple features with multiple classifiers.

Method	Evaluation (%)		
	Accuracy	Sensitivity	Specificity
SVM (LBP+HOG+GLCM) [17]	86.67	92.45	78.38
NB (morphological) [18]	81.11	69.81	97.30
Our method	91.11	94.34	86.49

**Table 5:** The accuracy (%) based on breast ultrasound image preprocessing.

Accuracy (%)	Features			
	LBP	HOG	GLCM	LBP + HOG+GLCM
Before preprocessing	81.11	80.00	71.11	82.22
After preprocessing	85.56	81.11	78.89	86.67

**Table 6:** The elapsed time before and after dimension reduction based on PCA.

	Time/s	
	Before dimension reduction	After dimension reduction
LBP+HOG+GLCM (SVM)	0.3601	0.0135

## Data Availability

The Breast Ultrasound Image data used to support the findings of this study were supplied by Quanzhou first hospital in Fujian, China, under license and so cannot be made freely available.
